# The Relationship between Burnout and Intention to Leave Work among Midwives: The Long-Lasting Impacts of COVID-19

**DOI:** 10.1155/2022/8608732

**Published:** 2022-08-09

**Authors:** Sahar Ahmadi, Azam Maleki

**Affiliations:** ^1^The Student Research Committee of Zanjan University of Medical Sciences, Zanjan, Iran; ^2^Social Determinants of Health Research Center, Zanjan University of Medical Sciences, Zanjan, Iran

## Abstract

**Objective:**

It is important to evaluate the long-term effects of the COVID-19 pandemic on the intention of midwives to leave their jobs. The study examined the relationship between burnout and the intent to leave work among midwives who worked at Ayatollah Mousavi Hospital of Zanjan, one year after the COVID-19 outbreak.

**Method:**

In a descriptive-analytical study, the intention of 88 midwives to leave their jobs was evaluated, one year after the outbreak of COVID-19 disease in 2021. The midwives were selected using convenience sampling methods. Data were collected using the Maslach burnout questionnaire and the Anticipated Turnover Scale (ATS). Data were analyzed with descriptive statistics, Chi-square test, Pearson correlation coefficient, and multiple linear regression model with the stepwise method at a 95% confidence level.

**Results:**

The mean intention to leave the job was 29.71 ± 6.75. Most of the midwives reported a moderate level of intention to leave the job (47.7%). There was a significant positive correlation between the intention to leave the job and all three components of burnout. The stepwise regression analyses indicated that emotional exhaustion (*β* = 0.344) and working rotational shifts (*β* = 0.276) were significant predictors of intent to leave the job.

**Conclusions:**

It can be concluded that the intention to leave the job of midwives was moderate. Given the relationship between emotional exhaustion and the intent to leave the job, interventions to increase the mental strength and resilience of midwives during the COVID-19 pandemic seem necessary.

## 1. Introduction

After the COVID-19 outbreak, the medical staff was on the frontline of the fight against the virus outbreak [1, 2]. They worked long hours under pressure with inadequate resources and facilities. They were burdened with additional risks associated with close interaction with COVID-19 patients [3]. At the start of the outbreak, 12.5% of 441 South Korean government employees consisting of nurses, physicians, and nonmedical staff including technicians and administrators intended to leave their job. The highest proportion of healthcare workers that indicated their intention to quit their job was physicians (14.6%). Additionally, 22% of frontline and 8.3% of those indirectly involved to COVID-19 patient care employees stated that they had thought about quitting their job due to the risk of infection. Among these, the nurses had frequently felt this (10.6%) [4]. Each occupation contains job demands and job resources that affect employee well-being and job satisfaction [5]. The impact of motivation and job stress on employee well-being and performance has been well described by the Job Demands-Resources (JD-R) model. Time pressure and workload are two main job demands which create a burnout condition that could seriously decrease the employees' well-being and finally cause low employee performance [6]. Organization support, skills progress, and autonomy as job resources could assist as a buffer in reaching organizational goals when job demands are high [7].

Burnout, absenteeism, and decreased productivity are consequences of work-related stress. Burnout is a syndrome characterized by emotional fatigue (a feeling of depleted mental capacity), depersonalization (devoid of emotions and excessive indifference to the service recipients), and feelings of lower personal accomplishment (a sense of diminished competence and professional success), which is more common among human service providers [8, 9]. The findings of Sohrabi et al. revealed that 28% of midwives working in hospitals and comprehensive health facilities in Sanandaj were struggling with emotional exhaustion, 33% were suffering from depersonalization, and 25.5% suffered from severe burnout failure. Job satisfaction, depersonalization, and failure at work were significantly associated with employment status [10]. The causes of burnout are complicated and comprise two distinct factors: environmental and individual factors. An example of a person-related element is personality qualities, motivation to choose a career, and self-expectations [11]. Burnout is one of the most salient factors in reducing efficiency and manpower loss, which is significant in two ways. To begin with, it harms people's mental health, causing physical symptoms and psychological problems such as headaches, digestive problems, risk of heart disease, marital issues, and even suicide. In addition, it decreases the quality of treatment provided to patients and leads to dissatisfaction with health services [10, 12, 13]. Consequently, burnout is associated with the intention to quit one's job [14]. Research conducted in Turkey during the COVID-19 outbreak revealed that midwives had 1.92 times higher risk of depression than nurses. There was also a 1.11 times higher likelihood of feeling depressed among midwives who experienced more emotional exhaustion [15]. Nonetheless, midwives serve as guardians of maternal and infant health at all levels of the healthcare system, including hospitals and community health centers [12, 16]. Also, during the COVID-19 outbreak, midwives serve as an auxiliary workforce without adequate training to deal with the crisis in COVID-19 wards, where COVID-19 patients are hospitalized [17]. The general assumption is that healthcare providers are experiencing higher levels of stress during the COVID-19 pandemic but the long-term effects of COVID-19 on various aspects of occupational health of employees have not been studied enough, especially in developing countries employees. Assessing midwives' health is critically important in determining whether a long-term pandemic will have an impact on their intention to leave the occupation. Therefore, this study was conducted to examine the relationship between burnout and the intent to leave the job among midwives who work at the Ayatollah Mousavi, a teaching hospital in Zanjan, one year after the COVID-19 outbreak.

## 2. Materials and Methods

### 2.1. Type of Study and Setting

A descriptive-analytical study was conducted to determine the intent to leave the job and its relationship with burnout among midwives working at Ayatollah Mousavi Teaching Hospital in Zanjan, a city in the northwest of Iran, one year after the COVID-19 disease outbreak in 2021. Ayatollah Mousavi Hospital in Zanjan is a quaternary health service. During the COVID-19 pandemic, patients are also triaged.

### 2.2. Participants and Sampling Method

The study population comprised of midwives who worked at the indicated hospital and were selected using the convenience sampling method. Inclusion criteria were a willingness to engage in the study and a minimum of six-month work experience in the hospital. A total of 100 midwives who worked at the hospital participated in the study, and, after considering the inclusion criteria, 88 individuals were qualified for the study.

### 2.3. Tools

The data collection tools included personal information, the Maslach burnout scale, and Anticipated Turnover Scale (ATS).

Demographic information included age, marital status, job experience, type of ward, type of employment, and shift type.

#### 2.3.1. Maslach Burnout Inventory (MBI)

This questionnaire is the most commonly used for measuring job burnout. It has 22 items that are scored in 7-point on a Likert scale ranging from never (zero) to every day (six). Twelve items of the scale are reverse scored. The questionnaire subscales include emotional exhaustion (9 items), depersonalization (5 items), and personal accomplishment (8 items). In the emotional exhaustion subscale (EE), a score of 17 and lower indicates a low degree of emotional exhaustion. A score of 18–29 and more than 30 demonstrates a moderate and high degree of emotional exhaustion, respectively. In the depersonalization subscale (DP), a score of 5 and lower demonstrates a low degree of depersonalization. A score of 6–11 and more than 12 demonstrates a moderate and high degree of depersonalization, respectively. In the personal accomplishment assessment subscale (PA), a score of 33 and lower demonstrates a low degree of personal accomplishment. A score of 34–39 and more than 40 demonstrates a moderate and high degree of personal accomplishment, respectively [18].

Moalemi evaluated the validity and reliability of the Persian version of the Maslach Burnout Inventory among Iranian nurses in two hospitals of Fasa University of Medical Sciences. They reported that the Persian version of MBI has sufficient validity and reliability. Also, Cronbach's alpha for emotional exhaustion subscale, depersonalization subscale, and personal accomplishment were 0.85, 0.76, and 0.71, respectively [19].

#### 2.3.2. Anticipated Turnover Scale (ATS)

The scale was originally developed in 1978 by Hinshaw and Atwood [20]. This questionnaire comprises 12 items that are scored on a 5-point Likert scale ranging from strongly agree to strongly disagree. The job turnover forecasting tool has an overall score between 12 and 60. Higher scores indicate a higher intention of turnover. Scores of 39 or higher (strongly), 29–39 (averagely), and 28 or less (weakly) predict the likelihood of leaving the job. The Persian version of ATS had very good psychometric properties in Mokarami's study among Iranian employees. Cronbach's alpha of the Persian version of ATS was 0.90 and the test-retest correlation coefficient was 0.87 [21]. In Hariri's et al. study, Cronbach's alpha coefficient of ATS was 0.82 among nurses [22].

### 2.4. Data Analysis Method

SPSS (version 16) was used for data analysis. The data were described using descriptive statistics. The Kolmogorov-Smirnov test was used to determine the data's normality. The data were normally distributed.

The Chi-square tests and Pearson correlation coefficient with a 95% level of confidence were used to examine the associations among variables. The Durbin-Watson statistic was used in this study to test for error independence, and the calculated value was 2.04. The Variance Inflation Factor (VIF) and collinearity tolerances are two collinearity diagnostic factors that can help us identify multicollinearity. In this study, collinearity and VIF were determined to be 0.97 and 1.02, respectively. Considering the aforementioned information, a stepwise multiple linear regression model with a 95% confidence level was used to identify the predictors of intent to leave the job.

## 3. Results

### 3.1. Demographic Characteristics

Our results indicate that the highest percentage of participants was between 26 and 35 years old (70.7%). Also, 61.4% of them were married, employed in a delivery room (45.5%), with less than five-year experience (48.9%), and rotational shift (86.4%) (Table 1).

### 3.2. Description of Burnout and Intention to Leave the Job

The average intent to leave the job score was 29.7 ± 6.75, emotional exhaustion was 16.81 ± 5.49, depersonalization was 5.02 ± 5.64, and personal accomplishment was 7.55 ± 12.86.

The frequency distribution of the intention to leave the job was 45.5% (*n* = 40) at the low intent level (ATS score 28 or less), 47.7% (*n* = 42) at the moderate intent level (ATS score 29–39), and 6.8 percentage (*n* = 6) at the high intent level (ATS score ≥40).

Regarding the depersonalization subscale (DP), 56.8% (50 people) reported low scores (score ≤ 5), 20.5% (18 people) reported moderate scores (score 6–11), and 22.7% (20 people) reported higher scores of depersonalizations (score ≥ 12). All of the participants (*n* = 88) reported high levels of personal accomplishment (PA) (score ≥ 40). Sixty-six persons (75%) reported a low degree of emotional exhaustion (EE). Seventeen persons (19.3%) and five persons (5.7%) reported a moderate degree of emotional exhaustion (EE).

### 3.3. The Relationship between Demographic Characteristics, Burnout, and the Intention to Leave the Job

The present study indicated that depersonalization had a statistically significant relationship with midwives' employment status (*p* = 0.035). Intention to leave the job had a statistically significant relationship with the type of hospital ward (*p* = 0.020) and shift work (*p* = 0.011). Thus, depersonalization was more prevalent among employed people who worked as part of a manpower plan and the intention to leave the job was more prevalent among midwives who worked on rotational shifts in the delivery ward, emergency department, and COVID-19 inpatient ward.

There was no statistically significant relationship between burnout subscales and other demographic characteristics. There was no statistically significant relationship between the intention to leave the job and other demographic characteristics (Table 1).

All demographic variables and the three dimensions of burnout were entered into the regression model. In a stepwise multiple linear regression model, after adjusting for gender, age, marital status, work experience, type of employment, and hospital ward, there was a relationship between emotional exhaustion and rotational shift work and the intention to leave the job. As a result, for every one-unit increase in emotional exhaustion, the intention to leave the job increases by 0.344. The chance for rotational shifts was 0.276 (Table 2).

A substantial positive correlation was observed between the burnout subscales and the intention to leave work (Table 3).

## 4. Discussion

### 4.1. Intention to Leave the Job

The purpose of the study was to examine the intention to leave work and its association with burnout among midwives who work at Zanjan Teaching Hospital, one year after the COVID-19 outbreak. According to the results of this study, approximately half of the participants showed a moderate intention to quit their jobs (47% moderate and 6.8% strong). In this context, Said et al. found that, in the first months following the COVID-19 pandemic in Egypt, 24.8% of nurses working in COVID-19 wards were willing to change the type of ward and 45.2% were willing to change the type of organization for employment. Intention to quit their jobs among nursing that worked in non-COVID-19 wards and COVID-19 wards was 10% and 34.3%, respectively. Also, 51% of nurses in COVID-19 units were dissatisfied with their job, compared to 42.9% in non-COVID-19 units. There was a significant correlation between the intention to quit a job and the number of working hours per week [23]. According to a study conducted in South Korea, 8.2% of hospital employees were willing to leave their jobs during the early stages of the COVID-19 pandemic, with nurses being the most willing to leave. The intention to quit was influenced substantially by the type of ward, perceived disease stress, and reported risk of death due to COVID-19 [4]. In a study by Liu et al., there was a moderate intention for nurses to abandon their careers at the onset of the COVID-19 outbreak in Wuhan, China. Resilience and perceived job benefits were directly correlated with the intention to leave a job [24]. Although there were differences in the study population, the intention to leave the job was higher than that reported in Said's study. Nonetheless, several predictive variables indicate a similar likelihood of leaving the job. The present study thus indicates that midwives who worked rotating shifts on delivery wards, emergency departments, and COVID-19 patient care departments had a higher propensity to leave their jobs. Observations suggest that the continuation of the COVID-19 pandemic poses a serious threat to the increasing intention to leave work in most countries, including Iran, and health policymakers should therefore pay attention to it.

### 4.2. Burnout

In the study, most participants felt a low level of depersonalization and low emotional exhaustion. Employees who worked under obligation to serve in public hospitals due to the use of free education facilities were more likely to experience being depersonalized due to the association between burnout rate and employment status. Based on a meta-analysis of 14 articles, the burnout rate for midwives was moderate (40%), which is consistent with the findings of the current study [25]. Another study of 27 articles from 17 countries showed that midwives in Australia, Canada, and Senegal suffered the highest burnout rates, while those in Finland and Norway suffered the least. Burnout has been connected to factors such as a heavy workload, significant environmental stress, insufficient job experience, and a lack of organizational support [26]. In contrast to a previous study, findings from the current study revealed a dramatic increase in midwives' sense of personal accomplishment since before the COVID-19 outbreak. The difference could be attributed to the prevalence of the COVID-19 and the stress and differences in the research environment. Feeling successful at work leads to increased self-confidence and mastery of tasks. Depersonalization leads to treating patients as if they are inanimate objects, with no regard or feeling. Experts believe that moderate to severe emotional exhaustion is caused by such personal stressors as role conflict, role ambiguity, overwork, interpersonal conflicts, and lack of independence, support, and reward, all of which contribute to mental exhaustion [27].

Rahmani et al. discovered that, during the COVID-19, the components of emotional weariness, depersonalization, and hospital staff personal accomplishment in Zahedan were 23.2%, 7.4%, and 57.5%, respectively. COVID-19 anxiety and burnout were also found to have a strong link. Young and single people with little work experience were more prone to burnout than others [28]. In terms of feelings of personal accomplishment, the present study's findings differed from those of the previous study, revealing that, during the COVID-19 pandemic, 19 midwives working in the hospital felt more unsuccessful than nurses working in other wards. The mismatch between employment status and salary earned with hard labor in the maternity wards, particularly the double stress caused by COVID-19 infection, appears to cause a sense of personal accomplishment in midwifery staff. As a result, it appears that planning to improve the job satisfaction of medical professionals, particularly midwives, during the COVID-19 outbreak, is important. There was a significant positive correlation between the burnout subscales and the propensity to quit in the present study.

Rotational shift work and emotional exhaustion also emerged as important factors in intention to leave a job. In 2014, Nikbakht et al. reported a similar result. According to their study, intention to leave the job in emergency departments occurred at a moderate rate, and there was a significant relationship between intention to leave the job and burnout [29]. Yörük and Güler in Turkey found a significant relationship between midwives' resilience and burnout during the COVID-19 pandemic [15]. Another study by Haji and Mohammadimehr in 2020 showed that, during the period of the COVID-19 pandemic, there was a positive relationship between job stress and the intention of Mahabad nurses to leave the service and a significant negative relationship with resilience [30]. Burnout is the opposite of resilience. Through resilience, people can overcome, transform, and even enjoy negative experiences. The study by Ghaderi et al. in 2018 showed that the intention of Sanandaj nurses to leave their jobs was unrelated to burnout [31]. Observed differences could be due to differences in the statistical population or the prevalence of COVID-19. Amid the COVID-19 pandemic, midwives played a crucial role in fighting the virus and protecting mothers and children. Midwives quitting during this period can impose additional burdens on organizations and increase burnout, resulting in lower quality maternal and child healthcare. Thus, improving the occupational health of midwives is recommended.

### 4.3. Limitation

The study did not measure the perceived stress or other organizational supports of midwives. Also, the study sample size was small, and the data were collected using a cross-sectional descriptive study method; doing cohort study with a large sample size and a long follow-up period is needed to obtain a better conclusion.

## 5. Conclusions

According to the study, we can conclude that there is a moderate intention to quit a job and a high level of personal accomplishment. Because of the connection between the intention to leave the job and the emotional exhaustion, it is necessary to build mental strength and resilience in midwives during the COVID-19 pandemic, especially in those who work in delivery rooms and have rotating shifts.

## Figures and Tables

**Table 1:** The relationship between burnout and the intention to leave the job with demographic characteristics (number = 88).

Variables	Participants (%)	Emotional exhaustion (%)			*p* value^*∗*^	Depersonalization (%)			*p* value^*∗*^	Personal/accomplishment	Intention to leave the job (%)			*p* value^*∗*^
		LOW	MOD	HIGH		LOW	MOD	HIGH		HIGH	LOW	MOD	HIGH	
*Marital status*														
Single	(38.6)	(33.3)	(58.8)	(40)	NS	(36)	(38.9)	(45)	NS	(38.6)	(37.5)	(40.5)	(33.3)	NS
Married	(61.4)	(66.7)	(41.7)	(60)		(64)	(61.1)	(55)		(61.4)	(62.5)	(59.5)	(66.7)	

*Work experience*														
1–5	(50.0)	(46.2)	(68.8)	(40)	NS	(42.9)	(66.7)	(52.6)	NS	(50)	(48.7)	(52.4)	(40)	NS
6–10	(14.0)	(18.5)	0	0		(14.3)	(16.7)	(10.5)		(14)	(12.8)	(16.7)	0	
11–20	(25.6)	(24.6)	(25)	(40)		(28.6)	(16.7)	(26.3)		(25.6)	(25.6)	(26.2)	(20)	
≥21	(10.5)	(10.8)	(6.3)	(20)		(14.3)	0	(10.5)		(10.4)	(12.8)	(4.8)	(40)	

*Age (year)*														
23–25	(20.5)	(19.7)	(17.6)	(40)	NS	(14)	(44.4)	(15)	NS	(20.5)	(15)	(26.2)	(16.7)	NS
26–35	(47.7)	(47)	(58.8)	(20)		(22)	(44.4)	(60)		(47.7)	(47.5)	(47.6)	(50)	
36–45	(22.7)	(24.2)	(17.6)	(20)		(30)	(11.1)	(15)		(22.7)	(25)	(23.8)	0	
≥46	(9.1)	(9.1)	(5.9)	(20)		(12)	0	(10)		(9.1)	(12.5)	(2.4)	(33.3)	

*Hospital ward*														
Emergency	(18.2)	(19.7)	(11.8)	(20)	NS	(18)	(16.7)	(20)	NS	(18.2)	(20)	(14.3)	(33.3)	0.020
Elective	(11.4)	(10.6)	(17.6)	0		(12)	(5.6)	(15)		(11.4)	(12.5)	(11.9)	0	
Delivery	(45.5)	(45.5)	(35.3)	(80)		(50)	(44.4)	(35)		(45.4)	(55)	(38.1)	(33.3)	
Postpartum	(19.3)	(21.2)	(17.6)	0		(16)	(33.3)	(15)		(19.3)	(10)	(31)	0	
COVID-19	(5.6)	(3)	(17.6)	0		(4)	0	(15)		(5.7)	(2.5)	(4.8)	(33.3)	

*Type of employment*														
Formal	(28.5)	(30.4)	(17.6)	(40)	NS	(36)	(5.6)	(30)	0.035	(28.4)	(35)	(21.4)	(33.3)	NS
Contractual	(12.5)	(16.7)	0	0		(16)	(16.7)	0		(12.5)	(17.5)	(9.5)	0	
Special contract	(17)	(13.6)	(19.4)	(20)		(14)	(11.1)	(30)		(17)	(10)	(19)	(50)	
Commitment	(42)	(39.4)	(52.9)	(40)		(34)	(66.7)	(40)		(42)	(37.5)	(50)	(16.7)	

*Type of shift working*														
Fixed	(13.6)	(16.7)	(5.9)	0	NS	(20)	(5.9)	(5)	NS	(13.6)	(25)	(2.4)	(16.7)	0.011
Rotational	(86.4)	(83.3)	(94.1)	(100)		(80)	(94.4)	(95)		(86.4)	(75)	(97.6)	(83.3)	

^*∗*^Chi-square test.

**Table 2:** A linear regression model of the intention to leave the job based on the stepwise method.

Variable	Beta	*R* ^2^	*β*	*p* value	95% CI	Tolerance	VIF
Emotional exhaustion	0.344	0.224	4.028	0.001	[−1.75, 6.31]	0.976	1.024
Type of shift working	0.276	0.224	2.668	0.006	[0.788, 4.547]	0.976	1.024

**Table 3:** Correlation of intention to leave the job with the subscale of burnout (*n* = 88).

	Intention to leave the job	Emotional exhaustion	Depersonalization	Personal/accomplishment
Intention to leave the job	1	—	—	—
Emotional exhaustion	*r* = 0.570^*∗*^	1	—	—
Depersonalization	*r* = 0.337^*∗*^	*r* = 0.630^*∗*^	1	—
Personal/accomplishment	*r* = 0.319^*∗*^	*r* = 0.434^*∗*^	*r* = 0.468^*∗*^	1

^*∗*^ *p* < 0.05.

## Data Availability

The data used to support the findings of the study can be obtained from the corresponding author upon request.

## List of Abbreviations

COVID-19: Coronavirus disease 2019
MBI: Maslach burnout inventory
EE: Emotional exhaustion
DP: Depersonalization
PA: Personal accomplishment
ATS: Anticipated Turnover Scale
VIF: Variance Inflation Factor.
